# Difficulties in the Treatment of Diabetic Foot and Research Progress of Combination of Traditional Chinese and Western Medicine

This article has been retracted.

**DOI:** 10.1155/2022/9449427

**Published:** 2022-08-11

**Authors:** Nie Wang, Yi Zhang

**Affiliations:** Shanghai Municipal Hospital of Traditional Chinese Medicine, Shanghai University of Traditional Chinese Medicine Preclinical Department, Chen's Surgery of Traditional Chinese Medicine, 200071, China

## Abstract

A diabetic foot is any disorder directly attributable to peripheral arterial disease (PAD) and/or the sensory neuropathies influencing the diabetic foot; it is a long-term (or “chronic”) complication of diabetes. Generally, it is a permanent (or “chronic”) comorbidity of diabetes. The swallowing of peripheral neuropathy and peripheral vascular disease leads to damage to the soft tissue, bone, and joint system of the foot. In addition, diabetic feet are also susceptible to infection, which can lead to lameness and even amputation. The management of the diabetic foot can be both challenging and chronic; it may comprise orthoses, surgery, antibacterial medication, and topical dressings. Traditional Chinese medicine (TCM) has a variety of methods for the treatment of diabetic foot with obvious advantages, which can be divided into internal treatment and external treatment of TCM. These treatments include external foot bath, fumigation and washing stains, internal administration of traditional Chinese medicine, syndrome differentiation and staging treatment, empirical prescription, self-made prescription, internal use of proprietary Chinese medicine, massage, acupuncture, and paste powder application, which have significant value in the prevention and treatment of diabetic foot. Some studies have shown that modern medicine combined with herbal therapy can significantly improve the prognosis of diabetic foot. Therefore, this study summarized the difficulties in the therapeutic approaches to diabetic foot and the recent research progress in combining Chinese and Western medicine in the treatment of diabetic foot.

## 1. Introduction

The incidence of diabetes has gradually increased. According to statistics, the incidence of diabetes in China has increased fourfold in the past 20 years. Long-term diabetes leads to a significant increase in the incidence of complications, as well as a higher rate of disability and mortality [1]. Compared with other developed countries, the related research on diabetic foot in China started relatively late. In the understanding of the disease, TCM emphasizes the combination of overall syndromic differentiation and local syndromic differentiation (the four diagnoses together) [2]. Moreover, TCM has a variety of approaches in the treatment of diabetic foot, which has obvious advantages. The modern medicine combined with herbal therapy can significantly improve the prognosis of diabetic foot. In addition, the related literatures have been reported.

## 2. Difficulties in the Treatment of Diabetic Foot

At present, the clinical managements of diabetic foot (DF) are divided into general, systemic, local, and surgical therapies. General treatment includes diet control, weight loss for overweight patients, self-care, and keeping warm. Systemic therapy can improve the overall status of patients and delay the progression of the disease by controlling the blood glucose level and applying anti-infective drugs, vasodilators, and neurotrophic drugs. Local treatment includes debridement, decompression, hyperbaric oxygen, and negative pressure, which can completely remove diabetic foot ulcers and gangrene, promoting wound healing [3]. Peripheral neuropathy usually starts from the distal toe to the knee. This indicates a possible early sign of peripheral neuropathy. As the condition progresses, the patient's motor, sensory, and autonomic nerves can be damaged. Once the feet lose its neuroprotective effect, it is easy to cause more harm. Most patients with diabetic foot are accompanied by diabetic peripheral neuropathy, mainly due to the motor nerve damage of diabetic foot, foot extensor, and flexor imbalance. In the advanced stages of diabetes, the muscles of the feet atrophy and the muscles lose their normal elasticity. DF is susceptible to bacterial infection, causing ulcers, cellulitis, and deep abscesses [4]. In addition, increased skin perfusion with autonomic nerve damage can lead to edema or atrophy and ulceration of the skin of the lower limbs.

The most common complication in patients with diabetes is peripheral neuropathy, which causes lower limb numbness, ant walking, insect crawling, fever, and electric shock-like sensation [5]. In patients where conservative treatment has failed, amputation is required to completely remove the necrotic tissue and prevent the disease from spreading. Revascularization therapy can restore the blood supply of patients, promote ulcer and amputation wound healing, and improve the quality of life of patients. Stem cell transplantation is the use of stem cell pluripotency. Through the secretion of many cytokines, vascular regeneration and extracellular matrix reconstruction can be promoted, which is conducive to the improvement and recovery of limb blood flow. However, most DF course cannot be effectively controlled the development through general and systemic treatments. Local treatment has some problems, such as incomplete debridement and ulcer recurrence. Long-term local treatment patients have poor compliance [6]. Modern medicine has been effective in the treatment of DF. However, the long treatment period and high costs for patients not only put great financial pressure on patients but also impose a greater burden on society and families. For DF with infection, long-term use of antibiotics will have drug resistance [7].

## 3. Understanding of DF in Traditional Chinese Medicine

According to Yuan Zhanying, “deficiency” and “blood stasis” are the pathogenesis of DF. “Deficiency” has three aspects, including qi deficiency, yin deficiency, blood deficiency. “Blood stasis” can be seen from five aspects, and phlegm and blood stasis, dampness and blood stasis, toxin and blood stasis, so vein obstruction, and qi deficiency and blood stasis are the total pathogenesis [8]. The book of Huang Di Nei Jing first recorded the content of “gangrene” and “carbuncle gangrene, which occurs in the toes of the foot, named Tuo carbuncle.” If it is dark, it will die without cure; if it is not black, it will not die. If you do not fail to cure it, you will die if you do not kill it urgently. “This is the earliest record of gangrene in traditional Chinese medical literature.” It is recorded in the theory of diabetes and storage of various diseases: “when the body fluid is exhausted, the meridians are astringent, and the meridians are astringent, then Ying and Wei are not good, and the hot qi stays, so it becomes carbuncle.”

“Eliminating thirst,” “gangrene,” and “blood arthralgia” are the understanding of DF in TCM. Its pathogenesis is based on qi-yin deficiency, while qi-blood meridian stasis and toxin block are the standard [9]. Zhang Xuewen believes that “Yin deficiency, dryness and heat, endogenous toxin” are the basic pathogenesis of DF [10]. Huang Xiangwu believes that the etiology of DF can be divided into two aspects, consisting of internal cause and external cause. Internal causes of prolonged illness can lead to an imbalance of qi and blood, Yin and Yang. Dampness and heat lead to deficiency of the tendons and veins, abnormal flow of qi and blood, and consequently stasis of blood in the lower limbs, while prolonged illness leads to occlusion of the veins, loss of nourishment of qi and blood in the tendons and skin, and decay into pus. From an external point of view, cold and dampness cannot be removed and the ligaments become inaccessible. Over time, this can lead to the affected limb becoming susceptible to necrosis due to loss of nourishment, further accelerating the formation of gangrene [11]. Xi Jiuyi believes that the pathogenesis of DF gangrene is mainly due to “dampness” and “heat,” which is in the fascia and tendons, so the pathological organs are to blame on the liver [12]. Professor LV Yanwei et al. pointed out that the etiology and pathogenesis of DF is mainly based on yin deficiency, resulting in deficiency of both qi and yin, endogenous dryness and heat, and later caused by exogenous dampness and toxin [13]. In addition, the occurrence of this disease is also related to improper diet and long-term smoking. Professor Wu Yiling put forward the theory of “choroid-vascular system disease,” pointing out that vascular endothelial dysfunction is related to the abnormal function of collaterals and qi stagnation, which is intrinsically consistent [14]. Diabetic patients suffer from long-term macrovascular and microangiopathy resulting in disruption of microcirculation in the foot. Therefore, it can be assumed that “venous stasis” is present throughout the disease process. Professor Pang He believes that the patients with this disease are weak in viscera and deficiency in body fluid, resulting in qi deficiency and blood stasis. Additionally, due to the invasion of external evil, evil toxin can enter the vein straightly, resulting in adverse blood qi [15].

## 4. Understanding of DF in Western Medicine

DF peripheral neuropathy is characterized by chronic, long-term low-degree inflammation. Inflammatory factors and a variety of immune factors are involved in the occurrence and development of DF peripheral neuropathy in the induction of insulin resistance. Further progression of DF may lead to darkening of the distal skin of the lower limbs, infection, and gangrene. The patients with severe foot infection and ulcers may show gangrene accompanied by diabetic neuropathy or lower limb angiopathy [2]. The main causes of DF are diabetic peripheral neuropathy, infection, and arteriopathy of lower extremities, which is from the viewpoint of Chinese DF Prevention and Treatment Guidelines (2019 edition) [16]. DF ulcer is a destructive component of diabetes progression [17]. Long-term extrusion and wearing of inappropriate shoes are also an inducement of DF, which accelerates the formation of DF to a certain extent. From the point of view of modern medicine, the related pathogenesis of DF is more complex [18]. On the one hand, diabetic patients have peripheral vascular lesions involving the blood vessels of the lower limbs, which can cause impaired blood supply to the feet. In the early stages, this mainly manifests itself as a weakened or even absent dorsalis pedis artery pulsation and a low foot temperature, which is easily overlooked by the patient. As the condition gradually worsens, the skin of the foot atrophies and thins, leading to ulcers and even gangrene, and eventually to the formation of DF. Second, the infection is an independent risk factor in DF ulcers. Considering that most diabetic patients are older and have poor immune system defenses, they are prone to infections [19]. DF is one of the serious chronic complications in patients with diabetes mellitus (DM). It is a local reflection of systemic lesions in the foot. It has a variety of manifestations; the most common form of which is foot ulcer. The clinical features of DF are early numbness, pains or absence of sensation in the limbs, chills, intermittent claudication, and resting pain [20].

## 5. Traditional Chinese Medicine Treatment of DF

### 5.1. Classification and Staging Treatment

Professor Dong Xiaopeng et al. divided DF into the following three syndromes, including Yin-cold and blood stasis syndrome, damp-heat toxin syndrome, and qi-blood deficiency syndrome [21]. These three subtypes can comprehensively guide clinical treatment. As Professor Lin Liying according to the relationship between the glory and loss of qi and blood and the rise and fall of evil in the development of DF, the treatment of DF is divided into three stages [22]. Professor Wang Xiuge proposed that the “three-stage syndrome differentiation and treatment of DF” should focus on clearing heat, promoting dampness and detoxification in the early stage, promoting blood circulation and removing blood stasis in the middle stage, and strengthening the body in the later stage [23]. According to Professor Zhou Yiye et al., the DF was divided into three stages, consisting of acute infection stage, remission stage, and recovery stage [24]. The patients in acute infection stage are able to treat with wet compress of wound combined with fumigation and washing of traditional Chinese medicine. In the remission stage, Ruyi Jinhuang powder was used externally on the wound and its surroundings. The results showed that staged intervention of external TCM treatment can promote the improvement of vascular endothelial function and enhance the ability of tissue regeneration, so it can cure or effectively relieve the symptoms of DF gangrene. DF was divided into five types, such as Yin deficiency and toxin exuberant type, damp-heat stagnation type, qi and blood deficiency remaining evil type, stasis toxin accumulation type, and qi deficiency and blood stasis type by Li Hongjun [25]. Among them, the type of yin deficiency and toxin is treated by clearing heat and detoxification, nourishing yin, and promoting blood circulation. Simiao Yongan decoction is used as the prescription. The treatment of dampness-heat stagnation type is clearing heat and promoting dampness, and activating blood circulation and detoxification. The selected prescription is Simiao Powder. In the treatment of deficiency of qi and blood, remaining evil is not clear, for replenishing qi and activating blood, supporting toxin and promoting muscle. The selected prescription is Tuoli Tuoyusan. The stasis and toxin accumulation type chooses the treatment of dredging collaterals and relieving pain, removing blood stasis and detoxification, and adding and subtracting Taohong Siwu decoction combined with Wuwei disinfection drink. Qi deficiency and blood stasis type is treated with nourishing qi and dredging the pulse, promoting blood circulation and removing blood stasis, and using Buyang Huanwu Decoction as the prescription. According to the different course of disease, DF was divided into two syndrome types, including deficiency of both qi and blood and excess of damp-heat and toxin by Zhao Yitong [26]. In the initial stage, it was the type of excess of dampness-heat and toxin, and the treatment was detoxification and detumescence, clearing heat and promoting dampness. Tangzu No. 1 was selected as self-made prescription. The middle and later stage was deficiency of both qi and blood. Acute onset, cold numbness, and other discomfort can be seen in a short period of time [27]. The recovery period is the later stage of DF, which is characterized by pale or yellowish complexion, often accompanied by fatigue and fatigue. The syndrome of deficiency of qi and blood is the dialectic of this period, which should be treated by Sijunzi decoction combined with Siwu decoction. This stage is the syndrome of blood stasis, which is treated by activating qi and activating blood. The improvement and remission period are mostly formed based on the acute stage, often visible cold fear cold, suffering from severe cold pain. This period is identified as a Yang deficiency and cold condensation syndrome and is treated with Yang and Tongdu.

### 5.2. Addition and Subtraction Treatment of Empirical Prescription

Professor Wang Mingqiang et al. showed that jiedu Tongmai recipe could greatly shorten the healing time of foot ulcer in patients with diabetes mellitus [28]. The internal administration of jiedu Tongmai recipe combined with MEBO is more beneficial to the healing of foot ulcers in patients with diabetes mellitus. Professor Chen Ma Zheng found silkworm feeding was used to remove the overlying degenerative and necrotic tissue of the wound during dressing change. The clinical efficacy of the two groups was compared after 7 days of treatment [29]. The overall effective rate of the treatment group was significantly higher than that of the control group. The treatment method of the experimental group was significantly better than that of the control group. Li Keke et al. showed that both the control group and the treatment group were treated with alprostadil and compound Danshen liquid, and the wound was regularly changed during the treatment [30]. The wound was washed with hydrogen peroxide and then dressed with compound Huanglian liquid dressing. Based on the above treatment, oral treatment of Yanggan Shengji decoction was added in the treatment group. The treatment lasted 1 to 6 courses. After the ulcer healed completely, the pills were made according to the above-mentioned decoction prescription and then continued oral administration for 4 to 6 courses. The results showed that the effective rate of the control group was significantly lower than that of the treatment group. Li Huizhi et al. selected Tangwanfang data from the 2021 master's thesis of Liaoning University of Traditional Chinese Medicine; 108 patients with urinary foot were divided into control group and treatment group [31]. The patients in the two groups were treated with routine Western medicine, and the treatment group was treated with Yiqi Huoluo Shengji decoction. After two courses of treatment, the total effective rate of the treatment group was significantly higher than that of the control group. The conduction velocities of tibial nerve, peroneal nerve, and ulnar nerve in the two groups after treatment were higher than those before treatment. In addition, the acceleration in the treatment group was more obvious.

### 5.3. Fumigation and Washing Treatment with Traditional Chinese Medicine

Lin Xia selected 120 cases and randomly divided them into the treatment group (*n* =64) and the control group (*n* =56). Before foot bath, the wound was disinfected with iodophor and washed with hydrogen peroxide or sterile saline, so that the necrotic tissue was effectively removed. The results showed that the total effective rate and wound area of the experimental group were better than those of the control group [32]. Du Lirong divided randomly 90 patients with grade 0 DF into two treatment groups (*n* =30) and a control group (*n* =30) [33]. The first group was treated with Qidan external washing prescription (Astragalus, Angelica sinensis, Guizhi, Evodia, Tongcao, Asarum, Dilong, Chuanwu Polygonum multiflorum, and Salvia miltiorrhiza). After treatment, it was found that Qidan external washing prescription could improve the symptom score, common peroneal nerve conduction velocity, and ankle-brachial index. Li Huai fumigated and washed patients with damp-heat toxin Shensheng diabetic foot ulcer with TCM (prescription for Poria cocos, Cortex Phellodendri, dandelion, rhubarb, diding, Radix Paeoniae rubra, Radix Atractylodis, Radix Achyranthes bidentata, Radix Sophorae flavescens, safflower, and through bone grass) [34]. After treatment, the total effective rate was 97.50% significantly higher than that in the control group 72.5%. The fumigation and washing method of traditional Chinese medicine are not difficult to operate and have little side effects, so it is worth recommending. 36 patients with grade 0 DF were treated with self-made Huoxue Tongluo foot bath prescription (Wuzao snake, safflower, Chuanxiong, Achyranthes bidentata, Angelica sinensis, chicken blood vine, and clinical addition and subtraction) by Xu Hongtao [35]. After 8 weeks of treatment, the total effective rate reached 86. 11%, and there was no adverse reaction. 40 patients with grade 0 DF were treated with TCM Fumai decoction (vinegar frankincense, vinegar myrrh, clove, safflower, chicken blood vine, salvia miltiorrhiza, aconite, Asarum, road pass, Polygonum cuspidatum root, licorice, Wulingzhi) [36]. After 3 weeks' treatment, the effective rate of the treatment group was 92.5% higher than that of the control group 64.2%. The effect of the treatment group was better than that of the control group. Xiao Yang suggested 43 patients with DF were randomly divided into control group (*n* =20) and experimental group (*n* =23) [37]. The results showed that the total therapeutic efficiency of the treatment group was significantly higher than that of the control group. 80 patients with DF were randomly divided into the control group and the experimental group by Yingying et al. [38]. Based on routine treatment of the control group, the treatment group used Tongbi decoction, which is a traditional Chinese medicine for promoting blood circulation, removing blood stasis, and dredging collaterals. The end of the course of treatment showed that the effective rate of the treatment was 92.19%, which was significantly higher than that of the control group (69.64%). The therapeutic effect was obvious.

### 5.4. Local Wound Treatment

Professor Wang Shuang et al. treated DF ulcers with Wuhuang Shengji ointment for external use [39]. Professor Chen believes that the disease is based on heat and qi deficiency, so rhubarb, Coptis chinensis, and Scutellaria baicalensis are used to clear heat and purge fire, break blood stasis and eliminate carbuncle, dryness, dampness, and detoxification, invigorate qi and invigorate spleen, support toxin, and promote muscle, Shengpu Huang cool blood in order to stop bleeding; all drugs play together to support upright and dispel evil, and treat both the symptoms and the root causes. 126 patients were randomly divided into the control group (*n* =61) and the treatment group (*n* =65) by Professor Xing Pengchao et al. [40]. Because of routine medical treatment, the patients in the treatment group were changed dressing every two days and were given Shenxiao Shengji Powder for external use. The results showed that the wound healing time and effective rate in the treatment group were significantly higher than those in the control group. 40 patients with diabetic foot were randomly divided into the experimental group and the control group [41]. The controls were treated with routine disinfection and debridement and the experimental group was treated with Baodu Shengji Powder based on the control group. After two courses of treatment, the results showed that the total effective rate of the experimental group was significantly higher than that of the control group. Selected 60 patients with DF were randomly divided into the control group and the experimental group [42]. The study showed that Puhua decoction reduced the level of serum AGEs and protected vascular endothelium to some extent. The release and synthesis of inflammatory factors are inhibited, promoting the establishment of peripheral vascular microcirculation in patients with diabetic foot gangrene, improving foot blood circulation, shortening ulcer wound healing time, and reducing the risk of amputation. Sixty-three patients with DF were randomly divided into the experimental group and the control group by Zheng Mingyue et al. [43]. The results showed that the wound area, granulation shape, wound exudation, and pain score in the experimental group were significantly higher than those in the control group. Xu Yani selected 40 DF patients and randomly divided them into the experimental group and the control group. After treatment, the blood glucose level of the treatment group was lower than that of the control group, and the wound healing time of the treatment group was significantly shorter than that of the control group. The method of nibbling debridement and changing dressing was used for debridement, and the purulent cavity was completely opened in order to facilitate drainage. The effect of this method is good; it is worth recommending [44].

### 5.5. Acupuncture Treatment

Tang Xiaohui et al. through meta-analysis concluded that moxibustion has a significant clinical effect in the treatment of diabetic foot [45]. According to the method of random number table, 80 patients with DF were divided into the experimental group and the control group [46]. The control group was treated with routine treatment, and the experimental group was treated with warm acupuncture on the basis of the control group. The acupoints of the patients were as follows: the acupoints of foot Taiyin and spleen meridian, foot sun, foot Shaoyang gallbladder meridian as the main acupoints. Another group of acupoints was Jiaqihai, Guanyuan, Taichong, Sanyinjiao, Zusanli, and Ashi. The total effective rate was 92.5% in the observation group and 65% in the routine group. The median nerve and common peroneal nerve conduction velocity in the experimental group was higher than that in the control group. 63 patients with DF gangrene (diagnosed by stage 0) were randomly divided into control group (*n* =32) and experimental group (*n* =31) by Niu Xuerui et al. [47]. Based on the control group, the experimental group took bilateral Zusanli, Fenglong, Yanglingquan, Chengshan, Feiyang, Hegu, Sanyinjiao, and other acupoints every day. After treatment, compared with the control group, the levels of hs-CRP and TNF-*α* in the treatment group reduced. Warm acupuncture has relatively few side effects, is easily accepted by patients, and can be widely used in clinical practice.

## 6. Progress in the Treatment of Integrated Traditional Chinese and Western Medicine

For the treatment of DF, it is very important to control blood sugar and improve the neurovascular condition of the affected area. Western medicine has great advantages in this respect. If there is wound infection, debridement and dressing change combined with related drugs are also the advantages of Western medicine. Traditional Chinese medicine pays attention to the overall concept of the disease, and the same is true for DF, which can cure both the symptoms and root causes of the disease. Combination of TCM and Western medicine can improve the therapeutic effect of DF and the prognosis of patients [48].

Guo Xian used the method of combination of traditional Chinese and Western medicine to treat DF; the main treatment measures are to control the level of blood sugar and hydrogen peroxide to clean the ulcer surface. Simiao Yong'an decoction for internal administration and Jinhuang ointment for external use, the curative effect is good. The ulcer surface is improved, and the quality of life is improved [49]. Luo Weidong was given Tongluo Huoxue Zhitong decoction (mainly Radix Astragali, Coptis chinensis, Flos Lonicerae, Radix scrophulariae, Radix angelicae Sinensis, Safflower, and Forsythia suspensa) based on diabetes diet, blood sugar control, anti-infection, and so on [50]. 98 patients with DF were randomly divided into the control group and the experimental group by Cheng Xuezhe et al. [51]. The control group was treated with routine debridement, and the experimental group was treated with Huashengji prescription combined with negative pressure closed drainage. After treatment, the total effective rate of the experimental group was significantly higher than that of the control group. The results show that Huashengji prescription combined with negative pressure closed drainage can improve the clinical effect of DF ulcer. Ninety patients with DF were randomly divided into 3 groups Yuan [52]. Group 1 was treated with nibbling debridement and ultrasonic debridement, followed by external application of pearl scald ointment; treatment group 2: after nibbling debridement and ultrasonic debridement, Vaseline gauze was treated with external dressing; and treatment group 3 was treated with pearl scald ointment after nibbling debridement and simulated ultrasonic debridement. The comparison of the total clinical effective rate of the three groups suggested that there were no shedding cases during the study period. At 7 and 14 days after treatment, the total effective rate in group 1 was higher than that in groups 2 and 3; after 14 days of treatment, the total effective rate in group 3 was higher than that in group 2. After 14 days of treatment, the wound healing rate in group 1 was higher than that in groups 2 and 3, and the wound healing rate in group 3 was higher than that in group 2.

62 patients with DF were randomly divided into the control group and the experimental group [53]. The control group was treated with transverse bone transfer of the tibia. The experimental group was treated with Sanhuang decoction based on the treatment of the control group. The results showed that the total effective rate of the experimental group was significantly higher than that of the control group, and the experimental group was significantly better than the control group in all indexes. 98 patients with DF were randomly divided into the experimental group and the control group [54]. The control group was treated with negative pressure closed drainage, and the experimental group was treated with Qidan Tongluo decoction on the basis of the control group to clear heat and detoxification, replenish qi, and nourish yin. The results showed that after 8 weeks of treatment, the experimental group was superior to the control group in the time of appearance of granulation tissue, time of ulcer healing, blood flow velocity, and internal diameter of dorsalis pedis artery. 50 patients with DF were randomly divided into control group and experimental group [55]. The control group was treated with debridement after anesthesia based on routine treatment, combined with continuous negative pressure closed drainage. The experimental group was treated with self-made Tangzu prescription based on the control group. The results showed that the scores of granulations, wound area, wound depth, and exudation in the experimental group after treatment were significantly lower than those before treatment and after treatment in the control group, suggesting that Tangzu prescription combined with negative pressure closure and drainage can accelerate wound recovery, reduce exudation, increase fresh granulation tissue, and accelerate wound healing. He Haofeng treated DF grades I ~ VI, and the control group was given low molecular weight heparin calcium, alprostadil intravenous drip, and oral cilostazole [56]. Based on the control group, the intervention group was treated with Tongluo gangue Yu recipe (peach kernel, safflower, Schisandra, etc.) combined with Huoxue Zhitong lotion (Bletilla striata, safflower, sappan wood, etc.) for 4 weeks. The clinical effective rate of the traditional Chinese medicine intervention group was higher than that of the control group. At the same time, combined with surgical debridement, nibbling debridement, whale swallowing debridement, and other applications can prevent further infection and promote the regeneration of granulation tissue.

A diabetic foot (DF) is any disorder directly attributable to peripheral arterial disease (PAD) and/or the sensory neuropathies influencing the DF; it is a long-term (or “chronic”) complication of diabetes. Generally, it is a permanent (or “chronic”) comorbidity of diabetes. However, it is undeniable that at present, there are still many key problems to be solved in the TCM treatment of DF. TCM syndrome differentiation, clinical stages, and other treatment standards are not unified. The specific evaluation criteria of clinical efficacy are inconsistent, and the questions reported in different studies are lack of comparability. There are not many prescriptions or proprietary medicines of traditional Chinese medicine commonly used in clinic. A few of experimental studies were carried out; however, the clinical research methods were unscientific and lack of convincing clinical observation data. The basic research on the specific mechanism of TCM in the treatment of diabetic foot needs to be strengthened. The simple application of traditional Chinese medicine and Western medicine has its own advantages and limitations. Moreover, the advantages and characteristics of TCM in the treatment of DF are fully demonstrated.

## 7. Summary

To sum up, some achievements have been made in the treatment of DF with traditional Chinese medicine, which shows the advantages of traditional Chinese medicine in the treatment of DF. In the process of treating DF ulcer with all kinds of TCM, the clinical treatment effect is improved, the course of disease is shortened, and the economic burden of patients is reduced. The treatment of DF by traditional Chinese medicine has a long history. Based on the idea of syndrome differentiation, the external treatment of traditional Chinese medicine shows a good clinical effect. The combination of internal and external Chinese medicine and modern medicine can shorten the course of treatment for patients, reduce recurrence, amputation, and mortality rates, and improve their long-term quality of life.

## Data Availability

The datasets used and analyzed during the current study are available from the corresponding author upon reasonable request.
